# Safety of Different Anesthesia Methods Combined with Intravenous Fast Channel Anesthesia in Lower Extremity Orthopedic Surgery of the Elderly

**DOI:** 10.1155/2021/9787879

**Published:** 2021-10-28

**Authors:** Peng Chen, Jia Yang, Dandan Hu, Xu Jing, Dajin Liu

**Affiliations:** ^1^Department of Anesthesiology, Suzhou Kowloon Hospital, Shanghai Jiao Tong University School of Medicine, Suzhou, Jiangsu 215021, China; ^2^Department of Anesthesiology, Huaian Hospital of Traditional Medicine, Huaian, Jiangsu 223001, China; ^3^Department of Anesthesiology, Huaian Jianghuai Hospital, Huaian, Jiangsu 223001, China; ^4^Department of Anesthesiology, The Affiliated Huaian Hospital of Xuzhou Medical University, Huaian, Jiangsu 223002, China

## Abstract

**Objective:**

To compare the safety of different anesthesia methods combined with intravenous fast channel anesthesia in elderly lower extremity surgery and the effect on postoperative outcome.

**Methods:**

A total of 106 elderly patients who underwent lower extremity orthopedic surgery in our hospital from February 2018 to February 2021 were selected and randomly divided into the control group (*n* = 53) and the observation group (*n* = 53) according to random number table. All patients received intravenous fast-track anesthesia. On this basis, the control group received spinal-epidural anesthesia, and the observation group received iliac fascial space block on the affected side combined with sciatic nerve block. The operation conditions, blood pressure and heart rate changes, awakening time, postoperative ICU admission rate, and complications were compared between the two groups.

**Results:**

There was no statistical difference in the success rate of one-time operation between the two groups (*P* > 0.05). The times of using analgesics and vasoactive drugs and the dosage of propofol in the observation group during the operation were lower than those in the control group, and the difference was statistically significant (*P* < 0.05). At T2, T3, and T4, the levels of HR, DBP, and SBP in the observation group were lower than those in the control group, and the difference was statistically significant (*P* < 0.05). After operation, the time of awakening, spontaneous breathing recovery, and extubation in the observation group were lower than those in the control group, and the difference were statistically significant (*P* < 0.05). The incidence of complications in the observation group was lower than that in the control group, the cognitive impairment was the most significant one in the incidence of single complication, and the difference was statistically significant (*P* < 0.05).

**Conclusion:**

Based on the combined intravenous fast channel anesthesia, the operation difficulty of the affected side iliac fascial space block combined with sciatic nerve block is the same as that of spinal-epidural anesthesia. It has a higher success rate of one operation, better analgesic and anesthetic effects during the operation, and little effect on blood flow of patients. It can maintain relatively stable heart rate and blood pressure and does not easily cause postoperative complications. Its safety is higher than that of spinal-epidural anesthesia.

## 1. Introduction

Due to the aggravation of population aging, the number of elderly patients undergoing lower limb orthopedic surgery is increasing. Many of these patients have many basic diseases, such as weak physical function, poor surgical tolerance, and high surgical risk [1, 2]. Therefore, how to ensure these patients to pass the perioperative period safely has become an urgent problem for anesthesiologists. Spinal-epidural anesthesia, nerve block, and intravenous fast-track anesthesia are all commonly used anesthesia methods for this kind of operation, each of which has its own advantages; however, there are various shortcomings in its separate application. With the development of propofol, an ultra-short-acting intravenous anesthetic, intravenous fast-track anesthesia has been widely used in cardiovascular and knee replacement operations [3, 4]. On the basis of applying intravenous fast-track anesthesia, combining with other anesthesia methods can significantly improve the operation effect, which has been widely recognized in clinic [5, 6]. Iliac fascial space block has been widely used in preoperative and postoperative analgesia and emergency medical treatment, its operation is simple, and its complications are less. Sciatic nerve block is one of the methods of local anesthesia, which can temporarily block the conduction function of the sciatic nerve. However, there are still relatively few research reports on the combination of anesthesia and anesthesia to achieve better safety. Therefore, this study explored the safety differences of different anesthesia methods combined with intravenous fast track in elderly lower limb orthopedic surgery. Specific reports are as follows.

## 2. Materials and Methods

### 2.1. Research Object

A total of 106 elderly patients who underwent lower extremity orthopedic surgery in our hospital from February 2018 to February 2021 were selected and randomly divided into the control group (*n* = 53) and the observation group (*n* = 53) according to random number table. Inclusion criteria: age ≥65 years; American Society of Anesthesiologists (ASA) rank II ∼ III (ASA classification was limited to a small range in order to minimize the impact of individual patient differences on this study); and cognitive function and mental state were normal before operation. Exclusion criteria: abnormal coagulation mechanism; immune system diseases; malignant tumors; surgical contraindications; and incomplete clinical data. The control group: 27 males and 26 females; age 65∼85years, average age (72.83 ± 5.92) years; 17 cases of ASA rank II and 36 cases of ASA rank III; 21 cases of lower limb internal fixation and total hip arthroplasty; 14 cases of replacement; 12 cases of artificial femoral head replacement; and 6 other cases. The observation group: 28 males and 25 females; age 65∼85 years, average age (73.95 ± 6.18) years; 17 cases of ASA rank II and 36 cases of ASA rank III; 17 cases of lower limb internal fixation and total hip arthroplasty; 15 cases of replacement; 14 cases of artificial femoral head replacement; and other 7 cases. There was no significant difference in general information between the two groups (*P* > 0.05). This study was approved by the ethics committee of our hospital.

### 2.2. Research Methods

#### 2.2.1. Anesthesia Method

After entering the operation room, upper limb venous access was opened and vital sign indexes were monitored routinely.

The control group: spinal-epidural anesthesia was given. Specific operation: lumbar puncture was performed at L3-L4, and 1.5 ml of 0.5% bupivacaine was injected, while 2% lidocaine was injected into the epidural space, and the anesthesia level was controlled below T10. After keeping the anesthesia position for 5 minutes, the position was changed.

The observation group: ultrasound-guided iliac fascial space block and sciatic nerve block were performed with 0.5% ropivacaine at a dose of 0.2 ml/kg. Specific positioning: the iliac fascial space block was performed 1 cm below the medial and lateral 1/3 of the line connecting the anterior superior iliac spine and pubic tubercle on the affected side. Three points including sacroiliac joint, greater trochanter of the femur, and sacral hiatus were marked, and a vertical line was made at the midpoint of the line connecting the former two points, and sciatic nerve block was performed at the intersection of the line connecting the former two points and the latter two points.

Intravenous fast channel anesthesia: all patients in the two groups were intravenously injected with 0.5–1 mg/kg propofol before skin incision and then continuously pumped with 0.06–1 mg/kg/min propofol until the end of the surgery, to maintain the bispectral index (BIS) value of 50–60.

In this study, according to the characteristics of our patient's condition, adrenaline, noradrenaline, and isoproterenol were used as vasoactive drugs during the operation.

#### 2.2.2. Observation Index

The following indicators between the two groups were compared: the operation conditions (including the success rate of one operation, analgesic drugs, vasoactive drugs, and propofol use during the operation); heart rate (HR), diastolic blood pressure (DBP), and systolic blood pressure (SBP) changes at different time points (including before anesthesia (T0), after anesthesia induction (T1), during tracheal intubation (T2), during surgery (T3), and during extubation (T4)); the time of awakening, spontaneous respiratory recovery and extubation; and postoperative complications (including cognitive impairment, infection, urinary retention, nausea, and vomiting).

### 2.3. Statistical Methods

The SPSS19.0 software was used for processing, measurement data are expressed by mean ± standard deviation (mean ± SD), and pairwise comparison is analyzed by the *t*-test. The enumeration data were compared among groups using the *χ2* test. *P* < 0.05 indicates that the difference is statistically significant.

## 3. Results

### 3.1. Comparison of Operation Conditions between the Two Groups

There was no statistical difference in the success rate of one-time operation between the two groups (*P* > 0.05). The times in the observation group during the operation were lower than those in the control group, and the difference was statistically significant (*P* < 0.05), as shown in Table 1.

### 3.2. Comparison of HR and Blood Pressure between the Two Groups

At T2, T3, and T4, the level of HR, DBP, and SBP in the observation group were lower than those in the control group, and the difference was statistically significant (*P* < 0.05), as shown in Figures 1–3.

### 3.3. Comparison of Time of Awakening, Spontaneous Respiratory Recovery, and Extubation between the Two Groups

After operation, the time of awakening, spontaneous breathing recovery, and extubation in the observation group were lower than those in the control group, and the difference was statistically significant. (*P* < 0.05), as shown in Figure 4.

### 3.4. Comparison of Postoperative Complications between the Two Groups

The incidence of complications in the observation group was lower than that in the control group, the cognitive impairment was the most significant one in the incidence of single complication, and the difference was statistically significant (*P* < 0.05), as shown in Table 2.

## 4. Discussion

Due to poor physical function of elderly patients, they are often complicated with various diseases, the reserve and compensation ability of important organs are significantly decreased, the perioperative hemodynamic fluctuations are large, the anesthesia risk is high, and there are many postoperative complications, which have seriously affected the operation situation, postoperative rehabilitation, and quality of life of the patients [7–9]. For this kind of patients, it is required not only to provide better anesthesia effect during operation but also to maintain the stability of hemodynamics to the maximum extent, so it is extremely important to choose appropriate anesthesia methods. Propofol is the most widely used intravenous anesthetic in clinic at present [10]. The peak time of blood concentration is only 2 min, and the efficacy of a single administration can be maintained for 5∼8 min. The half-life after continuous infusion is less than 25 min, and it wakes up quickly and completely without accumulation. Due to the emergence of propofol, intravenous fast-track anesthesia has been widely used in various operations, and its safety in elderly patients has been greatly improved compared with the past. However, there are still some shortcomings in its separate application [11]. At present, it is common to use intravenous fast track combined with other anesthesia methods in elderly patients undergoing lower limb orthopedic surgery, and it is of great significance to seek the best combined anesthesia scheme for elderly orthopedic surgery.

Fast-track intravenous anesthesia combined with spinal-epidural anesthesia or nerve block anesthesia is commonly used in clinical anesthesia. Spinal-epidural anesthesia can theoretically be used for all surgical anesthetics except those below the head and for postoperative analgesia, but its safety is unsatisfactory [12]. The results of this study showed that there was no statistical difference between the two groups in the one-time success rate of the operation, and all patients were successful at one time. The times of using analgesics and vasoactive drugs during the operation in the observation group and the dose of propofol consumed by intravenous fast-track anesthesia were lower than those in the control group. It shows that, with the development of ultrasound technology, the operation difficulty of nerve block anesthesia technology which was difficult to operate in the past is decreasing, which is equivalent to the one-time success rate of simple spinal-epidural anesthesia operation. In addition, nerve block anesthesia gives the patient a better anesthetic and analgesic effect, but has a minor effect on his vascular activity. Thus, the duration of analgesic and active drug application and the dose of propofol during intraoperative intravenous rapid anesthesia were lower than during spinal-epidural anesthesia [13, 14].

The stability of hemodynamics and the normal circulation function during operation are of great significance to ensure the safety of operation [15, 16]. The results of this study also show that the levels of HR, DBP, and SBP in the observation group are lower than those in the control group at T2, T3, and T4, which indicates that the blood flow changes little during operation and the fluctuation of vital signs is more stable after nerve block anesthesia in elderly patients, which can effectively guarantee the normal operation of the lower limbs. In addition, the awake time, spontaneous breathing recovery time, and extubation time in the observation group were lower than those in the control group. Compared with combined spinal-epidural anesthesia, nerve block can ensure the anesthetic effect during operation, and at the same time, it can save the anesthetic drugs at the same time, which has less influence on patients' bodies and quick recovery after operation and is safer for elderly patients. However, spinal-epidural anesthesia has a longer action time and wide drug diffusion, so it has a greater impact on the circulatory function and hemodynamics of the body [17]. In addition, it is also related to the higher dosage of propofol during operation if its anesthetic effect is compared with nerve block.

Elderly patients are prone to postoperative complications after lower limb orthopedic surgery, including cognitive dysfunction, pulmonary infection, gastrointestinal dysfunction, urinary retention, etc., and the occurrence of such complications is related to whether they can effectively block harmful stimulation during surgery and stress response and inflammatory response induced by surgical trauma [18]. Compared with spinal-epidural anesthesia, nerve block analgesia is more perfect, which can effectively block stress damage during operation, and it has no obvious effect on S2∼4, so it is not easy to lose bladder tension and lead to urinary retention. Comparing the postoperative complications of the two groups, the observation group was significantly lower than that of the control group, especially in cognitive dysfunction. There were five cases of cognitive dysfunction in the control group and no case in the observation group, suggesting that both iliac fascial space and sciatic nerve block are effective local anesthesia methods with high safety and good postoperative analgesic effect. The use of general anesthesia drugs during the operation was reduced, and it is safer for elderly patients.

## 5. Conclusions

Based on the combined intravenous fast channel anesthesia, the operation difficulty of the affected side iliac fascial space block combined with sciatic nerve block is the same as that of spinal-epidural anesthesia. It has a higher success rate of one operation, better analgesic and anesthetic effects during the operation, and little effect on blood flow of patients. It can maintain relatively stable heart rate and blood pressure and does not easily cause postoperative complications. Its safety is higher than that of spinal-epidural anesthesia.

## Figures and Tables

**Figure 1:** Comparison of HR between the two groups. *Note.* Compared with the control group, ^*∗*^*P* < 0.05.

**Figure 2:** Comparison of SBP between the two groups. *Note.* Compared with the control group, ^*∗*^*P* < 0.05.

**Figure 3:** Comparison of DBP between the two groups. *Note.* Compared with the control group, ^*∗*^*P* < 0.05.

**Figure 4:** Comparison of time of awakening, spontaneous respiratory recovery, and extubation between two groups.

**Table 1:** Comparison of operation conditions between the two groups (*n*, %).

Groups	One-time operation success rate	Times of using analgesics	Times of using vasoactive drug	Dosage of propofol (mg, mean ± SD)
Control group (*n* = 53)	53 (100)	5 (9.43)	4 (7.54)	52.12 ± 6.24
Observation group (*n* = 53)	53 (100)	1 (1.89)^*∗*^	0 (0)^*∗*^	35.67 ± 7.31^*∗*^

*Note.* Compared with the control group, ^*∗*^*P* < 0.05.

**Table 2:** Comparison of postoperative complications between the two groups (*n*, %).

Groups	Cognitive impairment	Infection	Urinary retention	Nausea	Vomiting	Incidence of complications
Control group (*n* = 53)	5	2	3	4	3	17 (32.08)
Observation group (*n* = 53)	0^*∗*^	1	0	2	2	5 (9.43)^*∗*^

*Note.* Compared with the control group, ^*∗*^*P* < 0.05.

## Data Availability

The data used and analyzed during the current study are available from the corresponding author.
